# A Versatile and Ubiquitous IoT-Based Smart Metabolic and Immune Monitoring System

This article has been retracted.

**DOI:** 10.1155/2022/9441357

**Published:** 2022-03-02

**Authors:** N. Arunkumar, V. Pandimurugan, M. S. Hema, H. Azath, S. Hariharasitaraman, M. Thilagaraj, Petchinathan Govindan

**Affiliations:** ^1^Department of Biomedical Engineering, Rathinam Technical Campus, Coimbatore-641021, India; ^2^School of Computing Science and Engineering, VIT Bhopal University, Kotri Kalan, Ashta, Near Indore Road, Bhopal, Madhya Pradesh 466114, India; ^3^Anurag University, School of Engineering, Department of Information Technology, Venkatapur, Ghatkesar Road, Hyderabad, Telangana-500088, India; ^4^Department of Electronics and Instrumentation Engineering, Karpagam College of Engineering, Coimbatore, India; ^5^Department of Electrical and Electronics Technology, Ethiopian Technical University, Addis Ababa, Ethiopia

## Abstract

In the present medical age, the focus on prevention and prediction is achieved using the medical internet of things. With a broad and complete framework, effective behavioral, environmental, and physiological criteria are necessary to govern the major healthcare sectors. Wearables play an essential role in personal health monitoring data measurement and processing. We wish to design a variable and flexible frame for broad parameter monitoring in accordance with the convenient mode of wearability. In this study, an innovative prototype with a handle and a modular IoT portal is designed for environmental surveillance. The prototype examines the most significant parameters of the surroundings. This strategy allows a bidirectional link between end users and medicine via the IoT gateway as an intermediate portal for users with IoT servers in real time. In addition, the doctor may configure the necessary parameters of measurements via the IoT portal and switch the sensors on the wearables as a real-time observer for the patient. Thus, based on goal analysis, patient situation, specifications, and requests, medications may define setup criteria for calculation. With regard to privacy, power use, and computation delays, we established this system's performance link for three common IoT healthcare circumstances. The simulation results show that this technique may minimize processing time by 25.34%, save energy level up to 72.25%, and boost the privacy level of the IoT medical device to 17.25% compared to the benchmark system.

## 1. Introduction

One of the main paradigms of networking is the internet of things (IoT), which spreads through a variety of claims, providing central access to and convergence of information [1]. Users and approved workers, such as medical practitioners, can have access to information according to the mission description for each person. Privacy and confidentiality, sensitive data security, and limited functionality are essential for healthcare [2]. IoT can connect the internet to a variety of sensors, cars, homes, and computers, enabling people to exchange statistics, evidence, and services.

This allows for information synthesis that can make the study, usability, and comfort of usage of data in submissions very important. IoT versatility has brought a number of new developments toward better data access and increased resource utilization and information sharing, among multiple causes, to boost complete data quality performance [3]. This is becoming possible thanks to advanced protocol networking technology innovations, high internet concentration, and consumer accessibility of large infrastructure. As a result, people are more concerned with consolidated acquisition and evaluation of data to save time and energy [4].

IoT's clever cities, intelligent houses, infrastructure, and economic surveillance are all critical issues. Healthcare has been one of the most critical issues, with accelerated industrialization, urbanization, and an ever-growing rate of senior citizens in Europe in recent years. The emphasis in healthcare is progressively moving from conventional methodologies, such as postdiagnostic therapy, to preventive and predictive health security. This pattern involves constant and systematic criteria for the monitoring of the individual's historical data from various fields of healthcare. This clinical internet of things is the foremost emphasis of the modern century of healthcare, after positive experiments with electronic (e-health) and mobile (m-health) [5].

An IoT-based medical platform is able to integrate and merge variables (on the server side) from various fields that can lead to protecting healthcare [6]. In 2016, the WHO stated that the second field in connection with healthcare that causes one in seven deaths was environmental criteria control involving physicochemical components. The larger and more advanced facilities most frequently follow these criteria. The facilities are only limited to being scattered by high operating costs, complicated calibration/recalibration, and advanced facilities in certain countries and towns. These stations, on the one hand, are not available anywhere for the environment, but on the other hand, they only provide an overview of the area [7]. The overview of medical healthcare is shown in Figure 1.

In this assessment, the environmental parameter category includes toxic/hazardous gases, sound, ultraviolet conditions, temperatures, moisture, and air pressure. Environmental sensitivity and physiological parameters are, therefore, two of the most critical areas for monitoring in the field of healthcare. In p2Health, the physiological and biochemical variables must be constantly tracked and customized. Several studies have identified adverse effects on the health status of environmental contaminants, particularly on patients with physiological parameters and vital indications [8].

Depending on the time of exposure, accumulation and quantity of toxins, and the clinical state of patients, the sensitivity of people with cardiac disease and cardiovascular disease to chemical air pollution is a major factor in their breathing rate and heart failure. The harmful effects of environmental contaminants are not only restricted to environmental criteria but also physical criteria. Physical environmental metrics classify the highest noise frequency, UV, weather, moisture, and intensity. Various studies have shown that noise has adverse effects on sleep efficiency [9]. It is given a higher weight in the case of people suffering from chronic illnesses. In monitoring patients with chronic obstructive pulmonary disease, it is critical, for example, to track the sound level as an environmental parameter.

The high level of sound will contribute to sleep disturbance and thereby affect the physiological state of the patient. Exposure to UV indexes above the threshold can also pose a health risk, particularly in patients with skin cancer and COPD. Similarly, air and moisture can create painful problems. Environmental toxins can have a direct or indirect impact on physiological parameters [10]. However, continuous control, data synchronization, and the analysis of the relationship between environmental and physiological parameters are a leap forward to studying the effects and weights of each parameter on the other. The effect may differ from one parameter to the next.

The internal and external actors should be carefully investigated and determined. For p2Health to incorporate mIoT, customizable control of the parameters is taken into account by means of effective wearables. Wireless network nodes are an inseparable IoT tier that contains multiple sensor nodes and is used for inter/intradata communication between nodes and levels. In addition, data from different topics of focus are measured, gathered, and transmitted, even inside the WSN. The composed information is communicated from the wireless sensor node to the receiver through an IoT entry to construct a database according to the physiological and environmental indicators of a person 24/7. The WSN can be extended to stretch the observation border, as appropriate, by a variety of nodes to various extents of medical concern.

All the key components of the WSN are wearable sensor nodes that are used for custom surveillance. The functional structure, with temperament proportion, breathing frequency, blood pressure, and physique illness, is most often used for the physique in the Tuner Frame Zone System. While in customized healthcare, the acquisition, observation and loading, and transfer of every information collection have already been demonstrated, and both physiological and environmental monitoring by means of a durable and effective approach remain unintegrated.

Furthermore, an effective wearable is lacking in the measuring of ambient parameters. Integration of data must be illustrated in an appropriate approach and framework using powerful strategies/models aimed at full and then customized observations of active healthcare constraints. This explanation is specified and then applied to the IoT, which must also be able to host a massive amount of data in real time. In addition, data acquisition should be modular to allow for bidirectional coordination between licensed staff and end users for required medical commands [11]. Smart interpretation of data should also be available through the algorithms applied.

### 1.1. The Main Objective of This Study

- We designed an IoT-based platform for a suitable wearability mode to comprehensively measure environmental, physiological, and behavioral factors.
- We offer a privacy-controlled download method to determine the discharge rate and local calculation rate for the data processing. This approach takes into account the present condition of the radio channel, the amount and importance of fresh healthcare sensing data, the estimated level, the bacterial level, and the computational work history to reduce computer delays, save on IoT device energy consumption, and enhance data protection.
- For medical analysis of parameter interactions, we integrate, synchronize, and process physiological and environmental parameters. This also involves seeing the data on the server.

### 1.2. Organization of the Study

In the introduction part are given the essential information about patient monitoring and how the IoT devices are most helpful for monitoring health in different aspects. The second part of this study is made of a detailed literature review for the existing works given for support of defining the problem. The third part of this study proposed a system and flow diagram of the framework of the immune monitoring system given with various parameters. The final part has the result and discussion with various analyses like temperature, utility, and respiration analysis like lot parameters compared and discussed.

## 2. Existing Work and Literature Review

IoT devices provide edge computing with lower energy use and computation delays, which enables computation-intensive and latency-sensitive applications. In order to lower the computer overhead for resource-limited mobile devices, the binary download as suggested picks a data transmission rate under a stochastic Wi-Fi channel with a single edge. In order to decrease energy usage under latency constraints on a multiuser grid, the partial reloading schema as presented employs time division and orthodontic frequency division. In order to lower the implementation latency and work error rate for the scenario with just a known server, the mobile offload strategy as presented leverages the Lyapunov optimization, provided that both the model transmission delay and the local implementation model are recognized.

Geman et al. presented that the attackers could be inquisitive about data security, such as where the user is located and how their IoT device is being used. Depending on how far the user is from the edge node, an edge device can learn about location information and IoT device usage patterns [1]. The privacy level is tied to the amount of sensing data that has to be sent and the offload rate. Koo and Hur mentioned and received the calculation reports from the device, the IoT device will first do the local processing, and after this, it will compare the current channel states with the previously saved channel states and data size to assess the privacy level that was obtained [12]. The IoT device incorporates techniques to purposely limit the offloading rate while the channel is healthy and to raise the offloading rate when the channel is unhealthy in order to safeguard user privacy. Privacy is shown in red, since the consumption pattern indicates the difference between the amount of real sensing data and the amount of offloading data that takes place when increased wireless channel strength is present. Whether the IoT device stays in certain places with severely degraded radio channels is shown as location privacy.

The effective approach within IoT needs the careful handling of many problems by the application of WBAN in healthcare for environmental and physiological control. Due to critical continuous surveillance, it is of serious concern to consume power for short-term WBAN connectivity and long-range data transfer from the mobile to the server. The most critical requirements are wearability mode, flexible approach to sensor acceptance, the possibility of expansion, data collection range, accessibility, and fusion. Another part of healthcare is the relationship between physiological and environmental indicators, which involves data examination and can only be seen by data analysis by appropriate algorithm decisions based on an individual's continuous supervision [1].

Dawood et al. elaborated, reflects on the most current and important work in the monitoring of environmental, behavioral, and environmental biological restrictions. All other works offered in this segment fulfill the needs of the IoT in this field. An IoT-based tropospheric monitoring network has been established in [13]. Kim et al. suggested using a platform designed for the evaluation of environmental parameters like fine dust and ozone in various modes of contact in the short/long term. Each unit conveys a container containing information, and the position and operating position through the LTE system in this ecological measurement stage. This parameter is calculated by an applied board, and the data are analyzed on the server. The number of planning boards was used to gather data to track various air pollutants on this site.

A description of the IoT-based multisensor platform for atmospheric parameters to monitor nitrous gas (NOx), carbon dioxide (CO), and ozone (O3), and temperature, moisture, and air compression is presumed. The stage can track environmental contaminants at a low concentration. This infrastructure is built around two shields, one of which contains the ATmega328. One shield is used for gas sensors; the other shield is used for temperature, moisture, and wind speed sensors. These are planned as a fixed framework for server transmission based on the Wi-Fi networking protocol. The machine is Linux based for data observation [2].

The IoT-based solution for indoor air quality surveillance (IAQM) based on ATmega1281 was stated in [6]. In this job, a complete IAQM device enables carbon dioxide calculation and sulfur dioxide (SO2). It presents nitrous gas (NO2), O3, chlorine (Cl2), and environmental relative humidity. The boards in a star configuration are linked to a gateway via Zigbee. The transitional port passes the data via Wi-Fi to the cloud. As a front-end amplifier aimed at the devices, the sensors use the LMP91000 chip. All devices remain situated and arranged for protection. That makes this platform a fixed boxing station, useful for domestic surveillance [3].

A low-cost wireless network of sensors is presented with a protocol and Wi-Fi for long-range data transmission. A framework for calculating particulate matter has been established in this study. While, due to its limited portability, this device is best suited for regular environmental monitoring, its extensive monitoring supports many of the environmental parameters. A wearable single-gas detector was conceived and implemented for volatile organic compounds based on a capacitive micromachined ultrasound transducer [4].

This watch has long-term surveillance, is low powered, and has a detection limit of 120 parts per trip. The data are transmitted via a low-power network to a mobile phone or Raspberry Pi 3 and through Wi-Fi from the gates to the cloud. Even though the wearability of the member nodes is efficient, the identification of the single aspect limits the scenarios for this instrument. P was approached with common sense as a handheld prototype of Olivier et al. This common-sense version tests many environmental toxins, namely, CO, NO, O3 gas sensors, and sensors monitoring light, humidity, and body position, and O3 gas sensors.

Data are transmitted from the prototype via a component from SparkFun to the smartphone. The information received is viewed on a mobile phone and transmitted via a Cinterion GPRS radio to a host server. These data are also presented and evaluated on the web server. There will be a customized CO2 and O3 ambient air detector. Ahamed et al. presented a strong calibration method that was considered in the production of W-air according to the ambient physical and textile parameters and breathing emissions. In order to estimate CO2, W-air uses the V OCs CCS811 sensor. The relationship between VOCs and CO2 in this prototype is expected to be solid [14].

The data obtained from each gas sensor were transferred to a smartphone for viewing at a time interval of five seconds and one minute, respectively. The IoT monitoring devices for environmental parameters are not confined to the above, but the methods proposed have been the most relevant and most recent research in this field. Various other works were discussed on indoor/outdoor environment control portable, mobile, and/or stationary equipment. This type of work addresses the issues like relative moisture and relative humidity raised in the preceding paragraph. The boards in a star configuration are linked to a gateway via Zigbee. The intermediate port passes the data via Wi-Fi to the cloud.

Sensors use flaws via front-end equipment to drive themselves. Because both sensors are arranged for protection, the device is useful as an immovable container position for domestic surveillance. In [15], a low-cost network of environmental sensors is demonstrated using a long-range data transfer protocol and Wi-Fi. An established platform for metal oxide (CO), (NO2), hydrogen (H2), ammonia (NH3), and methane is presented in this work for the calculation of particulates, light, colors, steam, UV light, and methane. While, due to its limited portability, this device is best suited for regular environmental monitoring, its extensive monitoring supports many of the environmental parameters.

In 2012, a wearable single-gas detector was developed and applied to organic volatile compounds on the basis of a capacitive micromachine ultrasonic transducer. This watch is built for sustained surveillance, is low powered, and has a LOD of 120 ppb. The data are sent in low-power mode to a smartphone or a Raspberry Pi 3. An advanced and portable medical surveillance system with multiple sensors is available. The chest is a control panel, ECG, temperature sensor, accelerometer, acceleration engine, light-emitting color changes, and pushbutton. It includes a chest-placed unit and a color-changing light-emitted diode. In reality, facial recognition and clinical specifications are tracked in this system along with location monitoring.

The user's health status can be monitored with the embedded vibration engine by identifying capacitive touch patterns. The incorporated color-shifting lead can be used to provide the holder with more insight into the present state of health. Finally, for emergencies, a pushbutton is issued. The e-health detector platform V2.0, Arduino, and Raspberry Pi are the first biometric shield. This system monitors the heartbeat, oxygen in the blood, air supply, body temperature, ECG, galvanic surface concentration, blood pressure, patient location, and muscle/electrochemicals. This device can measure pulse (EMG) [5].

Data are gathered through different alternatives: real-time patient status reporting and patient critical data transfer to a health department for assessment. Depending on the request, data transfer is enabled on the e-health sensor. A multisensor fusion approach is the foundation of the structural system. A service provider model is used in particular [16].

There are various challenges that must be correctly handled in order to propose an optimal solution for IoT with wearable implementation in healthcare for environmental and physiological monitoring. Due to important, ongoing monitoring, power consumption is a major issue for short-range communication in wearables and long-range data transfer from smartphones to the cloud. The most essential needs are wearability mode, flexibility in sensor adoption solutions, extension options and data collecting ranges, usability, and fusion. In medical care, the connection between physiological and environmental indicators requires data research and can only be proved by data analysis through adequate algorithm choices based on the continuous monitoring of a person.

## 3. Proposed System

A modular cellular data framework is presented to ensure preventive and workplace control of everyday practices in the healthcare IoT strategy. In order to track the ubiquitous criteria, portable handsets with comfortable wearability are used in comparison to the modular data collection strategy. To do this, a system has already been established for robust environmental parameter tracking. The solution is a mix of operating systems that specifically aims to offer functionality and design abilities for all the main facets of the platforms.

The following criteria and demands are discussed, given the high diversity of this area of study and the monitoring criteria focusing on physiological and psychological well-being and also on the effects of environmental parameters on the ground [17]. We spoke earlier about the need for continuous and systematic data tracking and processing in preventive medicine. Therefore, wearables must be wearable and compact and lightweight with a comfortable style of wearability. Research into the field of measuring accurate information in the real world, in particular, shows that measuring settings require less user control. For these components, special attention must be given to product selection and prototype design. The proposed system architecture is shown in Figure 2.

The wearable devices remain prudently selected after the accessible device rendering follows the stated guidelines for physiological and psychological parameter tracking. The proposed system is designed to fulfill these criteria in the environmental surveillance sector as a handheld prototype. These three research areas will effectively contribute to cardiovascular and workplace health by integrating them. A thorough monitoring of environmental and physiological criteria is required in order to obtain comprehensive monitoring of healthcare. Pervasive surveillance involves a range of sensors that lead to scale, weight, and thus to wearability growth.

In order to ensure that wearability is conveniently preserved, the architecture techniques in combination with efficient software creation have to be consistent with the careful hardware concept, in this respect, 3D space usage for the system and efficient goods [18]. A thorough and personal collection of parameter settings, based on the specified parameter sets and the assessment by approved staff, is needed for the broadness of investigational scenarios within the area of preventive and occupational monitoring. It should not be restricted to specific case studies or topic classes.

There is also a strong need for a broad range of operative capabilities to combine multiple devices and sensor nodes from different vendors. The modular information gathering system is called an IoT portal. In this model, the access point is modular to adapt to external designs and devices in various fields to supplement the data solution where required [19]. The usage techniques for all data sources and, therefore, both data routes are taken into consideration in one framework. This hybrid data usability has a considerable effect on the structure of the device as data are distributed.

The incorporation of different systems and their individual configuration is essential to allow the flexibility of such information bases in response to research issues. Furthermore, the single mixture and setup also impact proper process control readiness, which requires a stronger device structure. The practical definition follows a dispersed device method that disassociates basic purposes from the domain cloud toward the separate IoT entry, such as information contribution, information gathering, and processing. Therefore, its functionality centers on data collection and information control, including customer-related tracking process setup.

The highest level includes cloud systems with the internal p2Health-Cloud system and cloud solutions from external providers as gateways into indirectly open results. The p2Health-Cloud allows user-specific research to be planned, through the management of so-called measures, including data range, data delivery frequency, the appropriate formats, and so on. This configuration seeks unique sensor node solutions but sets the necessary parameters. The p2Health-Cloud is carried out in the field of data science, primarily by algorithms for the detection of potential major associations with the goal of elevating information synthesis and information analysis, and it takes into account data comparisons for both local and national reference databases [20].

The results will be given to the user and supervisor through a web interface where required. The second level is focused on personal mobile devices that act as IoT gateways and carry out measuring tasks. This involves connecting directly accessible data sources to the needed sensor node and indirectly accessible external cloud solutions, collecting and preparing data, and providing data for P2Health-Cloud as provided by the measurement procedures [21]. The collection of the appropriate data sources depends on the user's comprehensive monitoring of the registered sensor nodes and can be taken into account, if possible, as alternate nodes.

The gateway then becomes the data ability to concentrate on each inquiry and must adapt the data collection process to the collected data, transmitted data size, and power usage via a remote sensor node setup. At this step, the incorporation of external cloud solutions encompasses the information collected and is hence a major portion of the gateway message initiative [22]. The entry also handles wellbeing server decentralization and subordinate synthesis of data, including information synchronization, information configuration, and processing. The third stage contains the devices used by the handler in connection with the WBAN. At this stage, all entered data source classes are viewed while the implicitly available data sources react as flight recorders that do not provide any additional features.

The directly available sources, by comparison, also have network configurations that allow changing between various modes or allow comprehensive calculation and procedure structure configurations by way of allowing or average settings for warnings and data compression processing choices. This allows the measuring method to be optimized in relation to the requisite control and, if available, initial handling of information [23]. These sensor nodes most often include a level of the sensor that enables more sensors or modular substitution to be linked. This makes it easy to substitute or connect single sensor modules to the sensor node. Therefore, IoT devices may be customized for the relevant specific application with hardware.

IoT healthcare devices employ several sensors to monitor health data such as heart rate and ECG and to give healthcare recommendations, including telling users whether they should seek immediate medical attention and providing telehealth assistance [24]. The IoT gadget is powered by both the battery and the energy-harvesting module, which lets it locally complete compute jobs, remotely offload jobs, and store the remainder for later.

A newly generated sensed information from the IoT device over a particular time variable *l* for the data size *D*_1_^(*l*)^ would be handling the data received earlier of the buffer level value *D*_0_^(*l*)^. For simplicity, we are just omitting the time variable *l*. The computational partition method and the overall computation tasks have been divided into the captured data with the capacity *D*_1_^(*l*)^+ *D*_0_^(*l*)^ by *M* number of similar computational tasks [25]. The sensed information can be prioritized based upon the analytical model that can be represented as *Y*^*l*^.

Let the scenario be considered. The edge computer is receiving *Y*_1_^(*l*)^ from the IoT device-generated computational task through a communication pipeline with a power gain value of *g*^(*l*)^, that has been executed by the computer over the local module of *y*_0_^(*l*)^ in a computational speed over *g* bps. Also, during the process of the forthcoming computational tasks, the buffering of the processed tasks is like {*y*_0_^(*l*)^,  *y*_1_^(*l*)^}  ∈  {*m*_0_/*M*, *m*_1_/*M* }_0≤*m*_0_, *m*_1_≤*M*_. The communication channel's power value can be estimated through a model, that is,

(1) $$\begin{array}{c} P\left(g^{l+1}=\;n|g^{l}=m\right)=\;i_{nm}\;\;\forall m,n\in Ϝ, \end{array}$$

where *Ϝ* represents the collection of states present in the communication channel [26]. The total amount of energy that was consumed by the device has been represented as *ℵ* for handling every sensed information received from the sensor devices. The flow model of the proposed architecture is shown in Figure 3.

There is the possibility that an attacker who is inquisitive about the user's privacy, including the user's location and use behaviour, might get the results of the calculation sent to the IoT device via the edge device. For the sake of location privacy and usage pattern analysis, an edge device can track the activity of the IoT device by offloading history depending on the channel state of the user at different distances [27]. The privacy level is connected to the amount of sensor data that needs to be handled and the rate at which it may be transferred.

*Q* is the present state's discounted long-term utility or Q function, which is utilized to select the offloading policy. The present state *t*^(*l*)^ of the healthcare sensing data, radio channel status, anticipated renewable energy generated in the time slot, battery level of the IoT device, and computation history are taken into consideration while choosing the offloading policy [28]. This plan employs the channel model already established and simulates real-world events to help a person find the best course of action.

An IoT device analyzes the importance of healthcare data represented by *Y*^(*l*)^ and calculates the network maximum power to the edge device *g*^(*l*)^ while monitoring the data of size *D*_1_^(*l*)^ at the time slot *l*. Using this information, the IoT device calculates the harvested energy density *σ*^−*l*^ and watches the standard battery capacity of the IoT device *c*^(*l*)^. Also, the current state has been represented by *t*^(*l*)^={*D*_1_^(*l*)^, *Y*^(*l*)^, *g*^(*l*)^, *σ*^−*l*^, *D*_0_^(*l*)^, *c*^*l*^}. The complete set of states obtained can be collectively known as *B*.

To create an analogous number of calculation tasks, a fresh and buffered set of healthcare data, with size *D*_1_^(*l*)^+*D*_0_^(*l*)^ partitioned into *M* sets, is applied the computation division technique. We choose the transfer policy *y*^(*l*)^= [*y*_0_^(*l*)^, *y*_1_^(*l*)^] *ϵ* *B* to establish a compromise between exploration and exploitation by employing the greedy approach [29]. A further particular aspect of the offloading policy that optimizes *R*(*t*^(*l*)^, *y*) is that it is picked with a low probability compared to the other plausible offloading policies. It retains the remainder in the buffer, locally analyzes the data, and transfers one more of data *y*_1_^(*l*)^(*D*_1_^(*l*)^+*D*_0_^(*l*)^) to the IoT device.

The IoT device evaluates the relationship between the cost of sensed data and the amount of transferring information and also the current channel statuses to determine the privacy level that was reached once local processing is completed.

## 4. Results and Discussion

In customized healthcare, we aspire to track extended and ubiquitous criteria in comfortable wearability modes. We are working on identification and mitigation for the identification of earlier disease functions. Users, doctors, health criteria, and requirements were taken into consideration in the implementation of the solution. Thus, for a joint contribution to users and medicines, a scalable IoT portal has been introduced. In the one hand, medicinal products will identify functions, quantify parameters, talk to the consumer, track the data in real time, and adjust wearable to the appropriate research and therapeutic issues. The customers are not exclusively limited to particular vendors on the other hand.

The customer should choose solutions that are easy to adapt to programs. The data for transaction time are shown in Table 1. In reality, the handler ensures not have to be suitable in the workaround; nonetheless, instead, the IoT entry is compatible with the user. In specific, this approach can be used in professional conditions, particularly in communities where children are vulnerable to unsafe situations that could jeopardize their safety [30]. This involves miners, technicians/chemical workers, and heavy-duty manufacturing and construction workers/technicians. Physicians would have full access to a broad variety of parameters, which will lead to a wide variety of situations and important clinical correlations between parameters and diagnoses.

The transmission analysis is shown in Figure 4. Two sets of data are provided in support of the approach. The solution has been checked in the Life Science Automation Center in a chemical/analytical laboratory to ensure the reliability of measured data, real-time setup, sensor activation, server task specification, sufficient data transmission, and selection.

The subject was interested in a chemical reaction in a relatively noisy atmosphere while wearing Equivital, Fitbit, and Ubiqisense. The privacy level comparison and the energy consumption comparison are shown in Figures 5 and 6, respectively. This test was conducted under all safety and durability legislations. Only a small amount of data obtained is displayed here because of the limited space.

Here, air humidity, heat, NO2, and Ubiqisense noise, RR interval, breathing rate, pulse rates, and Equivital skin temperature were calculated. The data that are sent to the server demonstrate the sensitivity and correct functionality of the prototype for measuring, collecting, and transmitting data. The temperature analysis is shown in Figure 7.

The NO2 limit aimed at the model is from 3 to 49.2 ppm, and the LODs are 0.4 ppm. Nitrous acerbic was physically applied to Cu in this experiment, resulting in a chemical process and a release of NO2. This was achieved in several rounds of several dozes by the chemical technician. In high levels and a maximum reaction in low concentrates of 5 seconds, the reply and regeneration period of the device show the rapid response at once.

In this procedure, up to 21.8 ppm was detected in the spectrum of gas concentration. The sound level was simultaneously calculated. The utility comparison is shown in Figure 8. With 1 dB resolution, the system is limited from 32 to 85 dB.

The respiration analysis is shown in Figure 9. Noise during the test exceeded not more than 44 dB then, and in this respect, the usual noise was around 50 dB. These atmospheric conditions of the laboratory indicate air temperature and humidity. Vital signs were simultaneously tracked for the physiological parameters. The heart rate ranges between 74 bpm and 93 bpm. One of the essential indicators of a coordinated respiration rate followed a similar trend with a variable emotion amount and swing amount of 8 to 19 per minuscule. The measurement result of the R-wave peak, as the most important peak, is also calculated [31]. The time across every two peaks in RR is the time measured. From this parameter, the heart rate variability can be derived.

The temperature of the skin was eventually revealed. The data communication efficiency is shown in Figure 10. At the start of the procedure, the skin temperature of the technician is 26.3°C. At the conclusion of the test, the temperature has risen to 29.3°C. Both Fitbit parameters have been sent and synchronized to the server. They will be located in different server directories. The amount of information obtained below the constraint is shown by the various selection charges of the devices. During the 18-minute testing period, 2.250 noise samples (1.9 Hz), 0.985 moisture, and mid-air heat samples (1 Hz), and then 595 NO2 (0.5 Hz) samples were obtained for environmental monitoring.

The performance of the proposed system is shown in Figure 11. Similarly, 72 breathing rates, cardio activity, skin temperature, and 1.450 RR interval samples (1.34 Hz) were obtained (every 15 seconds). We also submitted the solution to many practical experiments where all the functionalities of the solution are checked. Consequences of around 6 hours and 55 minutes stand summarized here for results and interpretation.

The computational latency comparison is shown in Figure 12. The doctors specified the tasks and accordingly adjusted the unit in this experiment. In order to best assess the wearables, all measures of environmental-physiological activity have been setup to measure the largest possible spectrum. In summary, the customer before sleep was told to bring and act as his normal routing both goods and prototypes.

The findings show the user's tracking while sleeping. The final QVR comparison is shown in Figure 13. This indicates that the customer has a natural state during his night. There are some noise bursts; however, the effects immediately vanish, nonetheless and this happens on an insufficient solitary period and, therefore, can originate significant meddling. Heart frequency, respiratory rate, and slumber levels are seen and then analyzed. While the parameter analysis indicates the normal set, the individual has failed to deeply sleep. This study, however, aims to encourage the assessment, definition, proof of principle, and application of practical usefulness, and approaches and techniques instead of medical inquiries.

## 5. Conclusions

A health-monitoring IoT-powered healthcare device has been presented as a privacy-aware technique to estimate energy consumption, the privacy breach, and the IoT computation and energy expenditure in an offloading and local computing paradigm. This technique decides the offloading policy to use at the edge device from every time slot by considering the privacy level, energy usage, and processing delay. The suggested methodology incorporates a transfer learning technique, which is well known in the radio channel modeling community, and a learning architecture, both of which serve to enhance the system's learning capabilities for dynamic healthcare IoT systems. We implemented a robust, widespread, readily accessible, and easy-to-use IoT-based infrastructure for monitoring several types of environmental and physical parameters with the accuracy improvement in the transaction response of records by 26.75%, and the QVR value of the proposed structure reduced the inference and noise up to 70% in the framework. Additionally, we brought in a wrist-worn prototype with sensors that were only active in low-light environments. To support an effective end-to-end connection between the user and the physician, an IoT gateway, an intermediary hub between sensor nodes and servers, has been built. Instead of doing clinical studies, the focus was on the method validation, technological definition, and usability. In the future, the scope can include more parameters to the wearability model with the stripped antenna that can incorporate the framework for a better immune monitoring system in antiquated peoples.

## Figures and Tables

**Figure 1:** Overview of medical healthcare.

**Figure 2:** Proposed system architecture.

**Figure 3:** Flow model of the proposed architecture.

**Figure 4:** Transmission analysis.

**Figure 5:** Privacy level comparison.

**Figure 6:** Energy consumption comparison.

**Figure 7:** Temperature analysis.

**Figure 8:** Utility comparison.

**Figure 9:** Respiration analysis.

**Figure 10:** IoT data communication efficiency.

**Figure 11:** Performance of the proposed system.

**Figure 12:** Computational latency comparison.

**Figure 13:** QVR comparison.

**Table 1:** Transaction time (ms).

No. of EMRs	Masood et al.	Menaka et al.	Omtosho et al.	Proposed approach
100	20.43	20.13	23.50	18.54
200	20.63	22.50	25.67	19.02
300	23.18	24.02	26.33	21.78
400	24.50	27.43	26.92	21.50
500	24.34	27.24	27.00	22.33
600	25.47	31.72	23.50	23.00
700	26.33	32.33	25.67	25.93
800	28.78	35.77	30.38	27.33
900	30.01	37.00	31.81	27.89
1000	32.50	39.98	32.62	29.72

## Data Availability

The data used to support the findings of this study are available from the corresponding author upon request.
